The article "Thyme Oil and Thymol Counter Doxorubicin-Induced Hepatotoxicity via Modulation of Inflammation, Apoptosis, and Oxidative Stress" was retracted in 2024. Reasons: signs of a paper mill; suspected computer-generated content; unreliable results or conclusions; concerns about the data.

# Thyme Oil and Thymol Counter Doxorubicin-Induced Hepatotoxicity *via* Modulation of Inflammation, Apoptosis, and Oxidative Stress

**DOI:** 10.1155/2022/6702773

**Published:** 2022-02-07

**Authors:** Osama M. Ahmed, Sanaa R. Galaly, Mennah-Allah M. A. Mostafa, Emad M. Eed, Tarek M. Ali, Alzhraa M. Fahmy, Mohamed Y. Zaky

**Affiliations:** ^1^Physiology Division, Department of Zoology, Faculty of Science, Beni-Suef University, P.O. Box 62521, Beni-Suef, Egypt; ^2^Cell Biology and Histology Division, Department of Zoology, Faculty of Science, Beni-Suef University, P.O. Box 62521, Beni-Suef, Egypt; ^3^Department of Clinical Laboratories Sciences, College of Applied Medical Sciences, Taif University, P.O. Box 11099, Taif 21944, Saudi Arabia; ^4^Department of Physiology, College of Medicine, Taif University, P.O. Box 11099, Taif 21944, Saudi Arabia; ^5^Tropical Medicine and Infectious Diseases Department, Beni-Suef University Faculty of Medicine, Beni-Suef, Egypt; ^6^Department of Medical Oncology Affiliated Zhongshan Hospital of Dalian University, Dalian 116001, China

## Abstract

Doxorubicin (DOX) is an effective anticancer agent with a wide spectrum of activities. However, it has many adverse effects on various organs especially on the liver. Thymol, one of the major components of thyme oil, has biological properties that include anti-inflammatory and antioxidant activities. Thus, this study was designed to examine thyme oil and thymol for their ability to prevent doxorubicin-induced hepatotoxicity in Wistar rats. Hepatotoxicity was induced by an intraperitoneal injection of doxorubicin, at a dose of 2 mg/kg bw/week, for seven weeks. Doxorubicin-injected rats were supplemented with thyme oil and thymol at doses 250 and 100 mg/kg bw, respectively, four times/week by oral gavage for the same period. Treatment of rats with thyme oil and thymol reversed the high serum activities of AST, ALT, and ALP and total bilirubin, AFP, and CA19.9 levels, caused by doxorubicin. Thyme oil and thymol also reduced the high levels of TNF-*α* and the decreased levels of both albumin and IL-4. These agents ameliorated doxorubicin-induced elevation in hepatic lipid peroxidation and associated reduction in GSH content and GST and GPx activities. Further, the supplementation with thyme oil and thymol significantly augmented mRNA expression of the level of antiapoptotic protein Bcl-2 and significantly downregulated nuclear and cytoplasmic levels of the hepatic apoptotic mediator p53. Thus, thyme oil and thymol successfully counteracted doxorubicin-induced experimental hepatotoxicity via their anti-inflammatory, antioxidant, and antiapoptotic properties.

## 1. Introduction

The liver is a central organ in the human body, coordinating several key metabolic roles. Due to its unique position in the human body, the liver is exposed to a vast array of agents including alcohol and drugs, as well as pathogens that may able to impair its function [1]. The liver is intimately connected to inflammation for responding to harmful stimuli. However, sustained liver inflammation can induce liver fibrosis and cirrhosis or hepatocellular carcinoma (HCC). Inflammation and liver cancer may be linked through the inflammation-fibrosis-cancer axis [2]. HCC is common cause mortality worldwide [3, 4]. Chemotherapy is a key treatment for later stages to prevent recurrence after surgery [5].

Doxorubicin (DOX) is an effective anticancer agent with a wide spectrum of activities. The drug is frequently used to treat several types of cancer, both hematological and solid [6]. Unfortunately, DOX displays significant hepatotoxicity [7, 8], cardiotoxicity [9], nephrotoxicity [10, 11], and testicular toxicity [12]. Numerous mechanisms have been suggested for DOX-induced hepatotoxic and cardiotoxic side effects, including reactive oxygen species (ROS) and nitrogen species, lipid peroxidation (LPO), mitochondrial damage, and cellular toxicity [13, 14]. However, molecular mechanisms for DOX side effects await full elucidation. ROS produced by oxidative stress may damage deoxyribonucleic acid (DNA) [15]. ROS are efficiently eliminated by antioxidant enzymes that detoxify oxygen-free radicals. These enzymes include glutathione peroxidase (GPx), superoxide dismutase (SOD), and catalase (CAT) under normal physiological conditions [16].

DOX has been reported to have inflammatory actions by various publications. Ahmed et al. [8] revealed that DOX intraperitoneal injection once a week for six weeks induced a significant increase of serum level of tumor necrosis factor-*α* (TNF-*α*) and liver expression of nuclear factor-*κ*B (NF-*κ*B) and cyclooxygenase-2 (COX-2) together with a decrease of serum interleukin-4 (IL-4) level. Mahmoud et al. [17] also found a significant increase in serum TNF-*α* level and decrease in serum IL-4 level in DOX-injected rats.

DOX reportedly induces apoptosis by generating ROS and activating the apoptotic protein, protein 53 (p53) [18]. Currently, a worldwide tendency has developed toward traditional medicines and natural resources that are culturally acceptable and affordable. Natural products and plant constituents with anti-inflammatory and antioxidant activities protect against organ toxicity caused by DOX [19, 20]. Herbal medicines can augment drug chemosensitivity, diminish chemotherapy side effects, and thus help to prolong patient survival [21, 22]. Globally, traditionally used medicinal plants number between 10,000 and 53,000; however, few of these remedies have been biologically evaluated and require further exploration to characterize their therapeutic potential [23, 24]. The plant family, Laminaceae, includes basil, thyme, and rosemary. These plants produce potent natural antioxidants to treat several diseases and even cancers [25]. Additionally, thyme exhibits several beneficial properties, including antioxidative, antiseptic, carminative, and antimicrobial [26, 27]. The oil from thyme is an antibacterial, anticandidal, and antioxidant agent when used topically. These properties are responsible for their increasing popularity [28]. Among many constituents, thymol (2-isopropyl-5-methylphenol) is a dietary monoterpene phenol in substantial quantities in certain plants, such as *Thymus vulgaris* [29]. Thymol displays antimicrobial, antioxidant, and hepatoprotective effects [30, 31]. Thymol also has anti-inflammatory and antiapoptotic roles [32–34]. In conductance with the previous publications, the current study investigated the preventive impact of thyme oil and its major constituent, thymol, on liver injury, oxidative stress, inflammatory status, and apoptosis in DOX-intoxicated rats.

## 2. Material and Methods

### 2.1. Experimental Animals and Housing Conditions

Forty-eight male Wistar rats, weighing 120–150 gm, were used as experimental animals in this study. The Animal House Colony of the National Research Center (NRC), Cairo, Egypt, supplied experimental rats. Animals were maintained under surveillance for 2 weeks before the experiment to eliminate the possibility of intercurrent microbial infection. Rats were kept in polypropylene cages with well-aerated stainless steel covers at 25 ± 5°C and 12-hour daily natural light-dark cycles. Rats were allowed free access to water and a sufficient balanced standard pelleted diet *ad libitum*. All animal procedures complied with the institutional Experimental Animal Ethics Committee (EAEC) guidelines, Beni-Suef University, Egypt (Ethical Approval Number: BSU/FS/2014/10).

### 2.2. Chemicals and Drugs

DOX was purchased from Pharmacia Italia (Milan, Italy). Aspartate aminotransferase (AST), alanine aminotransferase (ALT), and alkaline phosphatase (ALP) kits were obtained from Biosystem S.A. (Spain). Serum albumin and total bilirubin kits were obtained from HUMAN Gesellschaft für Biochemica und Diagnostica mbH, Wiesbaden, Germany. Other used chemicals were ultrapure and were supplied from Sigma Chemical Company (MO, USA).

### 2.3. High-Performance Liquid Chromatography-Mass Spectrometry (HPLC-MS) Analysis

HPLC-MS analysis of thyme oil was conducted at the Faculty of Postgraduate Studies for Advanced Sciences (Central Laboratory), Beni-Suef University, Egypt, using an HPLC-MS system—Infinity 1260, Ailent Technologies, Germany—coupled with a Diode Array Detector (DAD). The stationary phase was C18, with dimensions of 250 × 4.6 nm, 5 *μ*m Microsorb-Varian. The mobile phase was an isocratic combination of acetonitrile (ACN):H_2_O (50 : 50) with a 1 mL/min flow rate. The column temperature was 25°C. Detection was at 274 nm. The injection volume for all samples and standard solutions was 10 *μ*L. Ten mg of oil was added to a volumetric flask and diluted to 100 mL with ACN:H_2_O (80 : 20) (100 *μ*g/mL). A stock solution of thymol (3 mg/mL) was prepared separately in ACN: H_2_O (80 : 20).

### 2.4. Thyme Oil and Thymol Preparation

Thyme oil was delivered by Purity Factory, Abu-Radi Industrial Area, Beni-Suef, Egypt. Thymol was obtained from Riedel-de-Haën AG, Seelze-Hannover Company, Germany. Thyme oil dose was prepared by dissolving 250 mg in 1% carboxymethyl cellulose solution (CMC). The dose of thymol was prepared by dissolving 100 mg in 1% CMC.

### 2.5. Experimental Protocol

Adult male Wistar rats were separated into four groups (6 animals/group) (Figure 1) as follows:

*Normal group*: the rats within this group received the equivalent volumes of the vehicles, which are 0.9% NaCl (1 mL/kg b.wt) by intraperitoneal injection one time/week and 1% CMC (5 mL/kg b.wt) every other day by oral gavage for 7 weeks

*DOX-injected control*: rats were intraperitoneally administrated DOX at 2 mg/kg b.wt one time/week for 7 weeks. Such group was also administered the equivalent volume of the vehicle (1% CMC kg b.wt) every other day by oral gavage for 7 weeks

*DOX-injected animals treated with thyme oil*: these rats were intraperitoneally administered DOX (2 mg/kg b.wt one time/week) and orally treated with 250 mg thyme oil/kg b.wt [35, 36] every other days by oral gavage for 7 weeks

*DOX-injected animals treated with thymol*: rats within this group were intraperitoneally administered DOX (2 mg/kg b.wt one time/week) and orally treated with 100 mg thymol/kg b.wt [35, 36] every other day for 7 weeks

### 2.6. Blood and Tissue Sampling

After seven weeks, rats were anesthetized by diethyl ether inhalation and then sacrificed. The blood samples were quickly taken from the right jugular vein. After decapitation and dissection, the livers were excised for biochemical, histopathological, immunohistochemical, and molecular investigations. After clotting, blood was centrifuged at 3000 rpm for 15 minutes. The clear sera were stored at -30°C. Liver tissue samples were homogenized in a sterile isotonic saline solution (0.9% NaCl, 10% (*w*/*v*)). Homogenates were centrifuged at 3000 rpm for 15 minutes, and the supernatants were maintained at -20°C. Also, pieces of the liver (3 mm^3^) were kept at -70°C for RT-PCR analysis.

### 2.7. Determination of Serum Levels of Parameters Related to Liver Function

Activities of AST and ALT in serum were measured consistent with the method of Gella et al. [37] using reagent kits from Biosystem S.A. (Spain). ALP activity in serum was determined with a colorimetric method [38] using reagent kits from the same source. Serum total bilirubin and albumin levels were also assessed colorimetrically as previously described by Jendrassik [39] and Doumas et al. [40], respectively, using reagent kits from HUMAN Gesellschaft für Biochemica und Diagnostica mbH, Wiesbaden, Germany.

### 2.8. Assay of Serum Levels of Tumor and Inflammatory Biomarkers

Alpha fetoprotein (AFP) and carbohydrate antigen (CA19.9), TNF-*α*, and IL-4 levels in serum were measured with ELISA kits, which were obtained from R&D systems (USA), according to the manufacturer's instructions.

### 2.9. Assay of Liver Lipid Peroxidation (LPO) and Antioxidants

Hepatic LPO and antioxidant biomarkers were assessed using chemicals purchased from Sigma Chemical Company (USA) and an Erba Chem 7-Clinical Chemistry Analyzer, Mannheim Gmbh, Germany. LPO was assessed as described by Yagi [41]. Reduced glutathione (GSH) content was assayed as described by Beutler et al. [42]. Glutathione-S-transferase (GST) and glutathione peroxidase (GPx) activities were assessed as described by Mannervik and Guthenberg [43] and Matkovics et al. [44], respectively.

### 2.10. Gene Expression Analysis

#### 2.10.1. RNA Isolation

RNA was separated from liver tissue as described by Chomczynski and Sacchi [45] using a GeneJET RNA purification kit, Thermo Fisher Scientific Inc., Rochester, New York (USA).

#### 2.10.2. One-Step Reverse Transcriptase-Polymerase Chain Reaction (RT-PCR) Assay for Gene Expression

A Thermo Scientific Verso 1-Step RT-PCR ReddyMix kit (Thermo Fisher Scientific Inc., Rochester, New York, USA) was used to analyze mRNA levels of B-cell lymphoma-2 (Bcl-2). Complementary DNA (cDNA) produced by reverse transcription was amplified using a Thermo Scientific Verso 1 Step RT-PCR ReddyMix. The final reaction volume was 50 *μ*L consisting of Verso Enzyme Mix (1 *μ*L), 2X 1-Step PCR ReddyMix (25 *μ*L), RT Enhancer (2.5 *μ*L), forward primer (10 *μ*M) (1 *μ*L), reverse primer (10 *μ*M) (1 *μ*L), template (RNA) (2 *μ*L), and nuclease-free water (17.5 *μ*L). Forward and reverse primers were obtained from Biosearch Technologies, South McDowell Blud, Petaluma, CA, USA. Primers for Bcl-2 gene were F: 5 ′GGGATGCCTTTGTGGAACTA3′ and R: 5 ′ CTCACTTGTGGCCCAGGTAT3′ [46]. Primers for the housekeeping gene, *β*-actin, were F: 5′ TCACCCTGAAGTACCCCATGGAG3′and R: 5 ′ TTGGCCTTGGGGTTCAGGGGG3′ [47].

Reaction tubes were placed on a double heated led thermocycler. Reactions included inactivation at 95°C for 2 min, followed by 35 cycles of denaturation for 20 sec at 95°C, 50–60°C for 30 sec, and 72°C for 1 minute. The final extension was at 72°C for 5 min. PCR products were separated using 1.5% agarose gel electrophoresis and stained with ethidium bromide in 1x Tris Borate Ethylenediaminetetraacetic acid (EDTA) buffer (TBE) of pH (8.3-8.5). The cDNA bands were observed with a gel documentation system. Gel images were analyzed by scanning densitometry (Gel Doc. Advanced ver 3.0), and relative expressions of Bcl-2, normalized to *β*-actin, were calculated.

### 2.11. Histopathological Investigation

Pieces of the liver from each rat were immediately excised, fixed in 10% neutral buffered formalin (NBF), and embedded in paraffin for 24 h. Embedded tissue was then transferred to 70% alcohol. Blocks were cut into 5 microns sections. Sections were stained with hematoxylin and eosin (H&E) [48] and examined with light microscopy. Histopathological scores were determined for each lesion in six animals of each group. The lesion score takes four levels. Zero (0) refers to absence of lesion, I refers to mild degree, II indicates moderate degree, and III denotes to severe degree.

### 2.12. Immunohistochemical Detection of p53

Liver samples, fixed in 10% NBF, were transferred to the Department of Pathology, National Cancer Institute, for processing, blocking, and sectioning. Five *μ*m sections were mounted on positively charged slides (Fisher Scientific, Pittsburgh, PA). The p53 reactivity was processed as described by previous our publications [49, 50]. Liver section images were captured using a digital camera (Leica, DM2500M Leica, Wetzlar, Germany). Examination and analysis of labeling used free software version ImageJ (1.51d) [51]. Integrated intensities were evaluated using the ImageJ software (in pixels) of positive reactions with p53.

### 2.13. Statistical Analysis

Data are presented as mean ± standard error (M ± SE). Data were analyzed by one-way analysis of variance (ANOVA) followed by LSD tests (PC-STAT, University of Georgia, 1985) to compare results among several groups [52]. Significant differences were considered at *p* < 0.05. Equation used in the calculation of percentage change is as follows: % change = ((Final − Initial)/Initial) × 100.

## 3. Results

### 3.1. HPLC-MS Analysis of Thyme Oil and Thymol

HPLC-MS analysis indicated in Figure 2 revealed the presence of Cyclohexane, bromo-; 2-Pentene, 4,4-dimethyl-, (E)-; Cyclohexane, bromo-; p-Cymene; o-Cymene; gamma.-Terpinene; Benzene, 2-methoxy-4-methyl-1-(1-methylethyl)-; Anethole; Thymol; 3-Methyl-4-isopropylphenol; Phenol; and 2-Methyl-5-(1-methylethyl). The thymol, 3-Methyl-4-isopropylphenol, p-Cymene, and o-Cymene derivatives are the most abundant.

### 3.2. Liver Biochemical Parameters

DOX injections for seven weeks caused a significant (*p* < 0.05) increase in serum ALT and AST activities and total bilirubin level. Conversely, DOX administration induced a significant (*p* < 0.05) decrease in albumin levels. Serum ALP activity was not significantly increased (*p* > 0.05).

Supplementation of DOX-injected rats with thyme oil induced a significant (*p* < 0.05) reduction in elevated serum AST, ALT, and ALP activities and total bilirubin level. In contrast, supplementation of DOX-injected rats with thyme oil displayed a detectable but nonsignificant (*p* > 0.05) increase in albumin levels. Administration of thymol to DOX-intoxicated rats induced a significant (*p* < 0.05) decrease in the elevated serum ALT and AST activities and total bilirubin level and a significant (*p* < 0.05) increase in lowered albumin levels. Moreover, thymol caused a remarkable but nonsignificant (*p* > 0.05) change in serum ALP activity compared with DOX-injected control animals. Thyme oil seemed more effective than thymol in reversing impacts on liver function, as indicated by detected biomarkers (Table 1). An exception was the effect of thymol on serum albumin level.

### 3.3. Tumor Markers in Serum

DOX administration caused a significant (*p* < 0.05) increase in serum levels of AFP and CA19.9. The treatment of DOX-intoxicated rats with thyme oil and thymol significantly (*p* < 0.05) countered these increases in AFP and CA19.9, reducing levels toward their normal values. Thyme oil was more potent than thymol (Table 2).

### 3.4. Serum TNF-*α* and IL-4 Levels

TNF-*α* serum level increased (*p* < 0.05) in DOX-injected rats and serum IL-4 level declined (*p* < 0.05). Treatment of these animals with thyme oil and thymol significantly reduced changes in serum levels (*p* < 0.05). Thyme oil was more effective (Table 3).

### 3.5. Liver Oxidative Stress and Antioxidants

DOX administration caused a significant (*p* < 0.05) increase in LPO in the liver. A significant (*p* < 0.05) reduction in the content of GSH and activities of GST and GPx, as compared to normal rats, was also observed. The treatment of DOX-intoxicated rats with thyme oil and thymol induced a significant (*p* < 0.05) reduction in the higher LPO levels and a significant reversal of the lowered content of GSH and activities of GST and GPx (Table 4).

### 3.6. Bcl-2 mRNA Expression

Administration of DOX for 7 weeks produced a highly significant (*p* < 0.01) reduction in Bcl-2 mRNA in rat liver. Treatment of DOX-injected rats with thyme oil and thymol produced a significant (*p* < 0.05) reversal of downregulated Bcl-2 mRNA expression. Thymol was more efficacious than thyme oil (Figure 3).

### 3.7. Histological Changes

Histological examination of normal rats' livers showed normal architecture of thin-walled central veins and normal hepatocytes with narrow blood spaces known as sinusoids (Figures 4(a) and 4(b)). DOX-intoxicated rats' livers (Figures 5(a)–5(e)) showed many pathological changes, including thickening of the hepatic capsule, cytoplasmic vacuolization of hepatocytes, fibroblastic proliferation in the portal tract, oval cell proliferation, focal hepatic necrosis, apoptotic hepatocytes, fibrosis surrounding bile ducts, newly formed small bile ducts, and strands of fibroblasts around hepatocytes. Supplementation of DOX-injected rats with thyme oil (Figure 6) and thymol (Figure 7) produced marked rescue of these pathological changes. Thyme oil showed notable liver histological architecture and integrity improvement, but slight activation of Kupffer cells remained (Figures 6(a) and 6(b)). After thymol treatment, congestion of hepatic sinusoids and mild sinusoidal leukocytosis, thickening of the hepatic capsule, and cytoplasmic vacuolization of hepatocytes, together with hydropic degeneration of hepatocytes were still visible (Figures 7(a) and 7(b)). The histopathological scores for each lesion were depicted in Table 5. The histopathological scores including thickening of the hepatic capsule, cytoplasmic vacuolization of hepatocytes and hydropic degeneration, fibroblastic proliferation in the portal tract and oval cell proliferation, focal hepatic necrosis and inflammation, apoptosis of hepatocytes, fibrosis around bile duct, and appearance of newly formed bile ductules and strands of fibroblasts around the hepatocytes were remarkably improved to a great extent as a result of treatment of doxorubicin-administered rats with thyme oil and thymol.

### 3.8. Immunohistochemical Staining for Liver p53

Liver p53 expression was detected *via* immunohistochemistry (Figure 8 and Table 6). Immunohistochemical staining revealed a weak reaction with p53, reflecting the low expression of this protein (Figures 8(a) and 8(b)). The livers from DOX-injected rats demonstrated strong positive staining for p53 protein, indicated by an intense brownish color (Figures 8(c) and 8(d)). After treatment with thyme oil (Figures 8(e) and 8(f)) or thymol (Figures 8(g) and 8(h)), color intensity decreased, indicating lower p53 levels. The effects of the two agents were similar.

## 4. Discussion

Chemotherapeutic drugs that are toxic to dividing cells are crucial for treating tumors [53]. Such drugs are toxic to tumor cells and affect normal cells [54]. DOX, an anthracycline antibiotic, is commonly used to treat human cancers but displays toxic effects on the liver [7, 8] and other organs, such as the kidney and the heart [9–11, 55]. Almost 40% of patients suffered from a liver injury after DOX treatment [56]. DOX causes an imbalance between free radicals and antioxidants. This imbalance leads to tissue injury primarily mediated by LPO and protein oxidation in tissues [57]. The current study shows the impact of DOX-induced hepatotoxicity manifested by a significant elevation in serum ALT, AST, and ALP activities and total bilirubin level, as well as a significant decrease in serum albumin. Elevated serum ALT and AST activities due to elevated leakage from necrotic and damaged hepatocytes due to DOX toxicity [58]. Similar results previously reported in a DOX-induced hepatotoxicity model [59, 60] indicated increments in the levels of AST and ALT in the serum of DOX-intoxicated rats. ALT is a well-studied parameter for detecting liver injury. Elevated levels of serum enzymes reflect cellular leakage and damage to the cell membranes in the liver [61]. Another key hepatic marker enzyme is ALP, an enzyme associated with membrane lipid in canalicular ducts. An increase in serum ALP activity indicates a biliary flow disturbance. Thus, extra and intrahepatic interference with the bile flow elevates ALP serum levels [62]. Serum concentration of bilirubin is specific for possible serious liver damage or biliary obstruction and indicates loss of liver function [63]. Albumin is an important blood component, and its serum level reflects synthetic liver capacity [64, 65]. Moreover, albumin is a carrier for many biological substances, e.g., essential fatty acid transport from adipose tissue to muscles. Consequently, decreased albumin levels suggest significant liver dysfunction [66].

DOX administration caused a significant increase in serum levels of AFP and CA19.9 compared to normal control animals. These changes are consistent with Ahmed et al. [8] who showed similar increases in AFP and CA19.9. High serum levels of these factors are important markers for the early stages of HCC [67]. DOX administration also produced significant upregulation of serum levels of TNF-*α* and significant downregulation of IL-4 levels [8]. Our TNF-*α* results agree with many investigators [68–70], who indicated that elevated serum TNF-*α* reflects a DOX-induced cascade of inflammatory events with increased production of proinflammatory cytokines. The significantly decreased IL-4 level after DOX-administration is consistent with Santos et al. [71]. IL-4 inhibits many functions of activated macrophages, including the secretion of reactive oxygen species and nitric oxide [72, 73].

Loss of apoptosis in tumor cells is the key event for cancer progression. Families of pro- and antiapoptotic genes regulate apoptosis. Proapoptotic genes of p53 and Bcl-2 associated X (Bax), and antiapoptotic gene of Bcl-2, are involved in regulating cellular proliferation and apoptosis [74, 75]. DOX-injection induced a significant decline in Bcl-2 mRNA expression and a substantial increase in the expression of p53, a critical proapoptotic protein upregulated in response to DNA damage. DOX may induce downregulation of Bcl-2 through ubiquitin-proteasomal degradation [76]. In contrast, DOX administration led to an increase in the Bcl-2:Bax ratio [77]. Bcl-2 and Bax appear to regulate apoptosis independently, but an *in vivo* competition exists between the two factors. Also, DOX treatment produced a significant increase in p53, consistent with our results. Bcl-2 family members have significant roles in liver homeostasis [7]. However, these proteins help suppress apoptosis in carcinogenesis rather than stimulate cell proliferation. DOX treatment downregulated Bcl-2 and suggested that ROS might act as signal molecules for DOX-induced cell death [78, 79]. Further, this process was still functional even in the absence of p53. The same study also suggested that the p53-dependent pathway can be stimulated *via* a p53-independent mechanism. Downregulation of Bcl-2 during DNA damage-enhanced apoptosis should be mediated at the transcription level by wild-type p53. However, similar changes in Bcl-2 levels occurred in DOX-treated p53 null Saos-2 cells.

Histopathological investigation of liver sections of DOX-intoxicated rats supports previous biochemical results. Liver sections exhibited thickening of the hepatic capsule, cytoplasmic vacuolization of hepatocytes, focal hepatic necrosis associated with inflammatory cell infiltration, fibroblast proliferation in the portal tract, fibrosis around bile duct, apoptosis of hepatocytes, and newly formed small bile ducts. The livers showed irregularly formed cell plates after DOX injection because of congestion of blood vessels, necrosis, and inflammatory cell infiltration [8, 58]. The livers of DOX-injected rats showed congestion of central veins, dilatation of sinusoids, inflammatory cells, cytoplasmic vacuolization, and pyknotic nuclei [80] in addition to focal inflammatory cells forming granulomas and periportal fibrotic lesions in the liver. Results from other publications are consistent with the present findings [58, 80, 81].

DOX may have various cellular targets. For example, targeting DNA may directly or indirectly result in Bcl-2 downregulation [82]. DOX triggered Bcl-2 downregulation, cytochrome C release from mitochondria, and activation of caspases 3 and 9 as well as p53 suggesting the involvement of a mitochondrially regulated intrinsic apoptosis pathway [82, 83]. The present results are consistent with these observations.

Deleterious biochemical and histological alterations in liver function and structure were associated with a marked elevation of liver LPO and a significant decrease in antioxidant (GSH) content and antioxidant enzymes (GPx and GST) activities. Several studies demonstrated the same findings. Hepatic damage after DOX exposure is likely due to the production of ROS and suppression of antioxidant defense mechanisms. Additionally, elevated LPO is a vital aspect of DOX liver toxicity [84, 85].

Phenolic compounds are potent antioxidants found in many plants and herbs, including *Thymus vulgaris.* These compounds can react with membrane phospholipid bilayers to peroxidation chain reactions initiated by ROS [86]. Thymol, the major *Thymus vulgaris* component, exhibits hepatoprotective properties [87]. The anti-inflammatory properties of thymus essential oil are at least partially responsible for its hepatoprotective effects [36]. Administration of thyme oil and thymol to DOX-intoxicated rats effectively ameliorated high serum activities of ALT, AST, and ALP and elevated total serum bilirubin level. Further, these agents reversed reduced albumin levels. These results are in concurrence with Grespan et al. [36]. In addition, thymol treatment rescued hepatocellular damage as evidenced by prevention of any increase in serum ALP, AST, or ALT activities [88]. Likewise, treating rats with thyme extract markedly reduced the elevated activities of ALT, AST, and ALP and the elevated level of total bilirubin in serum towards normal values, reflecting its efficacy for protecting against liver damage and demonstrating membrane stabilizing activity [89, 90].

Administration of thyme oil and thymol to DOX-injected rats reversed the altered levels of liver tumor markers AFP and CA19.9 in the present study. Consistently, thyme extract effectively restored AFP to normal levels in aflatoxin-induced liver injury [91].

Elevated levels of the proinflammatory cytokine, TNF-*α*, decreased while reduced levels of anti-inflammatory cytokine IL-4 increased in response to treatment of DOX-injected rats with thyme oil and thymol in the present study. This finding is completely consistent with El-Sayed et al. [69]. Further, the anti-inflammatory effects of thymol may be due to the suppression of TNF-*α* production [92, 93] (Figure 9). Anti-inflammatory effects of thyme oil reflect its main component, thymol [94]. Similarly, the anti-inflammatory properties of thyme extract are due to thymol content. Thymol inhibited human elastase activity, a marker of inflammatory disease [95]. Thymol improved the T helper cell-1 (Th1)/T helper cell-2 (Th2) ratio in mouse primary splenocytes, resulting in a reduction in the inflammatory response [96]. Conversely, thymol decreases IL-4 levels in pulmonary diseases. Thus, the anti-inflammatory effects of both thyme oil and thymol administered to DOX-intoxicated rats are due to suppression of Th1 and activation of Th2 [97, 98] (Figure 9).

DOX-injected rats treated with thyme oil and thymol upregulated hepatic Bcl-2 mRNA expression and downregulated p53 (Figure 9). Consistently, thymol decreased apoptosis by increasing the expression of Bcl-2 and decreasing expression of Bax in rats with experimentally induced myocardial infarct [33]. In addition to their essential role in intrinsic apoptosis, tumor suppressor protein, p53, activates the extrinsic pathway of apoptosis through the induction of various membrane proteins. P53 is a nuclear transcription factor and regulates cell cycle proteins' expression, blocks cell division progression, or stimulates apoptosis in response to severe DNA damage [99, 100] (Figure 9). Thyme extract upregulated Bcl-2 gene expression but decreased the level of p53, consistent with our findings [91]. Treatment with thymol increased Bcl-2 expression in tert-butyl hydroperoxide-induced oxidative stress in liver cells and significantly decreased the level of Bcl-2 protein expression [101]. Additionally, oral administration of the phenol isomer of thymol, carvacrol, at dose levels of 25, 50, and 100 mg/kg to rats for 2 weeks before dosing with thioacetamide resulted in a significant decrease in liver damage, liver sinusoidal congestion, and inflammatory cell migration [102]. Carvacrol treatment also markedly inhibited NF-*κ*B expression in a dose-dependent manner and increased the expression ratio of antiapoptotic Bcl-2 to proapoptotic Bax. Thus, the antiapoptotic effect of thyme oil in the present study is due to its two main components, thymol and carvacrol.

Thymol is a potent antioxidant and anticancer agent [103]. Thyme essential oil can show effects opposite to carcinogenesis due to the antioxidant activity of its constituents [28, 86, 104]. Conversely, both mRNA and protein levels of Bcl-2 were upregulated by hypoxia, while the phenol isomer of thymol, carvacrol, at concentration 600 *μ*M, suppressed Bcl-2 expression in hypoxic Human Pulmonary Artery Smooth Muscle Cells (PASMCs) [105], unlike our findings. Carvacrol downregulated mRNA and protein expression of Bcl-2 under hypoxia, leading to mitochondrial depolarization and apoptosis. Administration of thymol and its analog, carvacrol, for 14 days before DOX administration ameliorated heart dysfunction and oxidative stress parameters. Thus, thymol and carvacrol display cardio-protection that might be attributable to antioxidant, anti-inflammatory, and antiapoptotic activities [69].

The improvements in serum parameters related to liver function in the present study are associated with the amelioration of liver histological changes. Thyme oil appeared more potent than thymol. Histopathological examination showed slight activation of Kupffer cells after thyme oil treatment. Liver damage remaining after thymol treatment included congestion of hepatic sinusoids and mild sinusoidal leukocytosis, together with hydropic degeneration of hepatocytes, consistent with the publications of Grespan et al. [36] and Abd El Kader and Mohamed [89].

Improvement of liver function and integrity may be mediated *via* antioxidant properties of thyme oil and thymol (Figure 9). The high antioxidant activity of thymol, the main component of thyme oil, is attributed to phenolic hydroxyl groups that act as hydrogen donors to proxy radicals formed during the first step in lipid oxidation, thus retarding H_2_O_2_ and lipid peroxides' formation [106]. The present study showed a significant decrease in LPO and increases in GPx and GST activity and GSH level. Similarly, treatment of DOX-injected rats with thymol countered LPO elevation and restored the decreases in GSH content and GST activity [107]. Thymol enhanced the activity of antioxidant enzymes; GPx action was notable, inducing a highly significant decrease in MDA concentrations [108]. Thyme oil and thymol act as scavengers for ROS, thus protecting organs from cellular damage and necrosis (Figure 9). Their abilities to increase liver GSH content as well as GST and GPx activities provide substantial defense against ROS [90]. This defense, in turn, decreases oxidative stress and scavenges free radicals that cause stimulation of LPO and tissue damage [109].

## 5. Conclusion

Thyme oil and thymol counteract the hepatotoxicity of DOX; thyme oil appeared more efficacious than thymol. This preventive effect may be mediated by enhancing cellular antioxidant defenses and modulation of inflammation and apoptosis. However, clinical studies on humans are required to assess the efficacy and safety of thyme oil and thymol.

## Figures and Tables

**Figure 1:** Schematic figure showing experimental design and animal grouping.

**Figure 2:** HPLC-MS fingerprint of thyme oil. 1: Cyclohexane, bromo-; 2: 2-Pentene, 4,4-dimethyl-, (E)-; 3: Cyclohexane, bromo-; 4: p-Cymene; 5: o-Cymene; 6: gamma.-Terpinene; 7: Benzene, 2-methoxy-4-methyl-1-(1-methylethyl)-; 8: Anethole; 9: Thymol; 10: 3-Methyl-4-isopropylphenol; 11: Phenol; 12: 2-Methyl-5-(1-methylethyl).

**Figure 3:** Effects of thyme oil and thymol oral supplementation on liver mRNA expression of Bcl-2 relative to *β*-actin in DOX-injected rats. ^a^Significant as compared to normal at *p* < 0.05. ^b^Significant as compared to DOX-injected control at *p* < 0.05.

**Figure 4:** Photomicrographs (a, b) of liver sections of normal rats showing normal liver architecture formed of thin-walled central vein (CV), normal hepatocytes (H) arranged in hepatic strands, with narrow blood spaces between them known as sinusoids (S) and Kupffer cells (Kc) lining sinusoids (H & E ×400).

**Figure 5:** Photomicrographs of liver sections of DOX-injected group showing thickening of the hepatic capsule (HC) and cytoplasmic vacuolization of hepatocytes (V) (a), fibroblast proliferation (F) in the portal tract and oval cell proliferation (OV) as well as vacuolization of hepatocytes (V) (b), focal hepatic necrosis (NC) as well as apoptosis of hepatocytes (AP) (c), hypertrophied bile duct (BD) and appearance of newly formed bile ductules (nbd) (d), and fibroblast proliferation (F) around the hepatocytes (e) (H & E ×400).

**Figure 6:** Photomicrographs of liver sections of DOX-injected rats treated with thyme oil showing hydropic degeneration (HD) and dilated central vein (CV) (a), as well as slight activation of Kupffer cells (KC) (b) (H & E ×400).

**Figure 7:** Photomicrographs of liver sections of DOX-injected rats treated with thymol showing congestion of hepatic sinusoids (C) and mild sinusoidal leukocytosis (SL) (a), together with hydropic degeneration of hepatocytes (HD) (b) (H & E ×400).

**Figure 8:** Photomicrographs (a–h) of immunhistochemical stained liver sections. (a, b) Normal rat liver showing weak immunohistochemical reaction of p53 expression. (c, d) Liver sections of DOX-injected rats showing a strong positive immunohistochemical reaction of p53 expression marked by dense brown color in cytoplasm and nucleus of hepatocytes. (e, f) Liver sections of DOX-injected rats treated with thyme oil showing a substantial decrease in the expression of p53. (g, h) Liver sections of DOX-injected rat treated with thymol showing a substantial decrease in the expression of p53.

**Figure 9:** Schematic diagram showing the effects of thyme oil and thymol on TNF*α*, IL-4, p53, and Bcl-2 for modulating inflammation, apoptosis, and oxidative stress.

**Table 1:** Effects of thyme oil and thymol oral supplementation on liver function biomarkers in serum of DOX-injected rats.

Groups	Parameters									
	ALT (U/L)	% change	AST (U/L)	% change	ALP (U/L)	% change	Total bilirubin (mg/dl)	% change	Albumin (g/dl)	% change
Normal	49.33 ± 2.72	—	187.67 ± 5.98	—	201.33 ± 10.19	—	0.56 ± 0.03	—	3.75 ± 0.25	—
DOX-injected control	62.50 ± 2.79^a^	+26.70	212.00 ± 4.93^a^	+12.96	233.33 ± 8.13	+15.89	0.70 ± 0.05^a^	+25.00	2.17 ± 0.11^b^	-42.13
DOX-injected group treated with thyme oil	40.00 ± 2.02^b^	-36.00	185.00 ± 7.79^b^	-12.74	173.17 ± 11.28^b^	-25.78	0.51 ± 0.04^b^	-27.14	2.42 ± 0.20^a^	+11.52
DOX-injected group treated with thymol	52.33 ± 5.25^b^	-16.27	189.17 ± 7.24^b^	-10.77	248.00 ± 15.56^a^	+6.29	0.57 ± 0.03^b^	-18.57	3.08 ± 0.37^b^	+41.94
F-prob.	*p* < 0.01		*p* < 0.05		*p* < 0.001		*p* < 0.05		*p* < 0.01	
LSD at the 5% level	10.09		19.40		34.26		0.12		0.74	
LSD at the 1% level	13.76		26.46		46.73		0.16		1.01	

Data are represented as mean ± standard error (M ± SE) of six rats. ^a^Significant as compared to normal at *p* < 0.05. ^b^Significant as compared to DOX-injected control at *p* < 0.05. Percentage changes were computed by comparing DOX-injected group with normal and DOX-injected groups treated with thyme oil and thymol with DOX-injected control.

**Table 2:** Effects of thyme oil and thymol oral supplementation on tumor markers AFP and CA19.9 in serum of DOX-injected rats.

Groups	Parameters			
	AFP (ng/mL)	% change	CA19.9 (U/mL)	% change
Normal	0.37 ± 0.04	—	117.32 ± 2.35	—
DOX-injected control	1.12 ± 0.12^a^	+202.70	386.90 ± 36.10^a^	+229.78
DOX-injected group treated with thyme oil	0.64 ± 0.07^ab^	-42.86	164.30 ± 5.96^b^	-57.53
DOX-injected group treated with thymol	0.67 ± 0.08^ab^	-40.18	190.67 ± 14.04^ab^	-50.72
F-prob.	*p* < 0.001		*p* < 0.001	
LSD at the 5%	0.24		57.91	
LSD at the 1%	0.33		78.98	

Data are represented as M ± SE of six rats. ^a^Significant as compared to normal at *p* < 0.05. ^b^Significant as compared to DOX-injected control at *p* < 0.05. Percentage changes were computed by comparing DOX-injected control with normal and DOX-injected groups treated with thyme oil and thymol with DOX-injected control.

**Table 3:** Effects of thyme oil and thymol oral supplementation on serum TNF-*α* and IL-4 levels of DOX-injected rats.

Groups	Parameters			
	TNF-*α* (pg/mL)	% change	IL-4 (pg/mL)	% change
Normal	31.43 ± 1.28	—	105.47 ± 3.47	—
DOX-injected control	102.80 ± 7.76^a^	+227.08	51.44 ± 4.97^a^	-51.23
DOX-injected group treated with thyme oil	49.80 ± 4.83^ab^	-51.56	87.03 ± 5.70^ab^	+69.19
DOX-injected group treated with thymol	77.13 ± 7.73^ab^	-24.97	82.53 ± 6.38^ab^	+60.44
F-prob.	*p* < 0.001		*p* < 0.001	
LSD at the 5%	15.47		17.76	
LSD at the 1%	21.10		24.22	

Data are represented as M ± SE of six rats. ^a^Significant as compared to normal at *p* < 0.05. ^b^Significant as compared to DOX-injected control at *p* < 0.05. Percentage changes were computed by comparing DOX-injected control with normal and DOX-injected groups treated with thyme oil and thymol with DOX-injected control.

**Table 4:** Effects of thyme oil and thymol oral supplementation on LPO and various antioxidants in the liver of DOX-injected rats.

Groups	Parameters							
	LPO in the liver (nmole MDA/100 mg tissue/hr)	% change	Liver GSH content (nmole/100 mg tissue)	% change	Liver GST activity (mU/100 mg tissue)	% change	Liver GPx activity (U/100 mg tissue)	% change
Normal	50.04 ± 1.74		45.50 ± 5.00	—	55.73 ± 1.92^a^	—	162.08 ± 2.96	—
DOX-injected control	60.14 ± 1.28^a^	+20.18	23.74 ± 1.78^a^	-47.82	41.70 ± 1.71^a^	-25.17	140.10 ± 4.68^a^	-13.56
DOX-injected group treated with thyme oil	43.05 ± 3.93^b^	-28.42	37.17 ± 3.34^b^	+56.57	48.59 ± 2.07^ab^	+16.52	152.99 ± 4.25^b^	+9.20
DOX-injected group treated with thymol	41.54 ± 4.78^b^	-30.93	37.50 ± 3.23^b^	+57.96	51.94 ± 2.25^b^	+24.56	156.71 ± 4.56^b^	+11.86
F-prob.	*p* < 0.01		*p* < 0.01		*p* < 0.001		*p* < 0.01	
LSD at the 5% level	9.67		10.40		5.89		12.30	
LSD at the 1% level	13.18		14.18		8.03		16.77	

Data are represented as M ± SE of six rats. ^a^Significant as compared to normal at *p* < 0.05. ^b^Significant as compared to DOX-injected control at *p* < 0.05. Percentage changes were computed by comparing DOX-injected control with normal and DOX-injected groups treated with thyme oil and thymol with DOX-injected control.

**Table 5:** Histological lesion scores of the liver in normal control, DOX-administered group, and DOX-administered groups supplemented with DOX-injected rats with thyme oil and thymol.

Histological changes	Score	Normal control	DOX	DOX + thymol oil	DOX+ thymol
Thickening of the hepatic capsule	0	6 (100%)	1 (16.7%)	6 (100%)	4 (66.6%)
	I	—	1 (16.7%)	—	2 (33.3%)
	II	—	2 (33.3%)	—	—
	III	—	2 (33.3%)	—	—

Cytoplasmic vacuolization of hepatocytes and hydropic degeneration	0	6 (100%)	—	2 (33.3%)	2 (33.3%)
	I	—	1 (16.7%)	2 (33.3%)	1 (16.7%)
	II	—	2 (33.3%)	1 (16.7%)	1 (16.7%)
	III	—	3 (50%)	1 (16.7%)	2 (33.3%)

Fibroblastic proliferation in the portal tract and oval cell proliferation	0	6 (100%)	1 (16.7%)	6 (100%)	6 (100%)
	I	—	1 (16.7%)	—	—
	II	—	2 (33.3%)	—	—
	III	—	2 (33.3%)	—	—

Focal hepatic necrosis and inflammation	0	6 (100%)	—	6 (100%)	5 (83.3%)
	I	—	2 (33.3%)	—	1 (16.7%)
	II	—	2 (33.3%)	—	—
	III	—	2 (33.3%)	—	—

Apoptosis of hepatocytes	0	5 (83.3%)	1 (16.7%)	5 (83.3%)	5 (83.3%)
	I	1 (16.7%)	1 (16.7%)	1 (16.7%)	1 (16.7%)
	II	—	2 (16.7%)	—	—
	III	—	2 (33.3%)	—	—

Fibrosis around bile duct	0	6 (100%)	1 (16.7%)	5 (83.3%)	4 (66.6%)
	I	—	2 (33.3%)	1 (16.7%)	2 (33.3%)
	II	—	3 (50%)	—	—
	III	—	1 (16.7%)	—	—

Appearance of newly formed bile ductules and strands of fibroblasts around the hepatocytes	0	6 (100%)	—	4 (66.6%)	5 (83.3%)
	I	—	1 (16.7%)	2 (33.3%)	1 (16.7%)
	II	—	2 (33.3%)	—	—
	III	—	3 (50%)	—	—

0: absence of lesion; I: mild; II: moderate; III: severe. The number of animals in each group is 6. The % in parentheses is the percent of animals in each grade.

**Table 6:** Immunohistochemical staining intensity (pixels) for p53 in liver normal control, DOX, DOX + Thyme oil, and DOX+ Thymol groups.

Groups	Parameters	
	p53 × 10^3^	% change
Normal	3.35 ± 0.12	—
DOX-injected control	617.05 ± 1.10^a^	18319.40
DOX-injected group treated with thyme oil	2.77 ± 0.02^b^	-99.55
DOX-injected group treated with thymol	2.80 ± 0.03^b^	-99.55
F-probability	*p* < 0.001	
LSD at the 5% level	1.64	
LSD at the 1% level	2.24	

Data are expressed as M ± SE of three rats. ^a^Significant as compared to normal at *p* < 0.05. ^b^Significant as compared to DOX-injected control at *p* < 0.05. Percentage changes were computed by comparing DOX-injected control with normal and DOX-injected groups treated with thyme oil and thymol with DOX-injected control.

## Data Availability

Data are available and accessible under reasonable request.
